# Stopping the Revolving Door: Reducing 30-Day Psychiatric Readmissions With Post-discharge Telephone Calls

This article has been retracted.

**DOI:** 10.7759/cureus.21174

**Published:** 2022-01-12

**Authors:** Antonia Phillip, Garrett Rossi, Roshi DeSilva

**Affiliations:** 1 Psychiatry, AtlantiCare Regional Medical Center, Galloway Township, USA

**Keywords:** psychiatry and mental health, inpatient care, public psychiatry, system based research and organized psychiatry, discharge criteria, rate of readmission, hospital readmission rate, cost reduction

## Abstract

This prospective study sought to determine the effect of a post-discharge telephone call on 30-day readmission rates at a short-term inpatient psychiatric facility. The patient population consisted of English-speaking adults in the age group of 18-65 years with a high school education or higher and met involuntary commitment criteria. Participants received a telephone call 72 hours after discharge using a standard script. Three hundred and forty-two patients completed the study. A Pearson Chi-Square test was used to analyze the data. We used an alpha level of 0.05 for all statistical tests. Total readmissions were reduced by 3.4% (p = 0.004) during the time of the intervention when compared to patients receiving standard care the year prior. During the intervention period, the average readmission rate was 9.9% (95%CI 5.9-12.1%). We conclude that systematic telephone follow-up has the potential to reduce 30-day readmission rates for inpatient psychiatric facilities.

## Introduction

Individuals with mental illness must be integrated back into the community after relatively short hospital stays. Many patients are discharged with inadequate social and financial support, which results in a revolving door between the community and inpatient facility. The period immediately following discharge from an inpatient psychiatric facility remains a time of vulnerability for many patients. Some challenges patients face after discharge include a lack of psychoeducation, long waits to access outpatient services, and difficulties with medication administration (e.g. long-acting injectables) or adherence [1]. Studies indicate that adverse events during the post-discharge period can lead to early readmission [1]. Targeting interventions for the period immediately following discharge may reduce readmission risk. There is considerable interest in the role of post-discharge phone calls as a means of reducing readmission risk [2]. Post-discharge phone calls aim to identify potential gaps in care that occur after discharge and allow for reinforcement of discharge instructions and follow-up plans.

Other medical specialties include a post-discharge call as a part of their intervention bundle for all patients discharged from the hospital [3]. The benefit of post-discharge calls as a stand-alone intervention has produced inconclusive results based on literature review [2]. However, many of the studies that evaluated the impact of telephone follow-up were limited by small sample sizes and heavily screened populations, which limit the effectiveness of the intervention [4]. To date, there are few studies published in the literature that address the use of post-discharge telephone calls in patients leaving an inpatient psychiatric care facility. Using data from a large community-based inpatient population, we aimed to evaluate the utility of all-cause 30-day readmission rates with post-discharge telephone follow-up. 

## Materials and methods

The study was approved by the Geisinger Institutional Review Board (GIRB) (Approval # 2019-0315).

Site and study population

This study took place in a community short-term care facility (STCF) hospital in Atlantic County, New Jersey, USA. The duration of the study was from July 2019 to July 2020. The catchment area includes two additional counties, Salem and Cape May. The facility consists of 34 total beds split evenly between male and female patients. The majority of the beds are reserved for patients who meet commitment criteria with two beds being reserved for voluntary admissions. Participants were recruited during inpatient admission. Those patients who met the criteria and volunteered for the study were considered the intervention group. Three hundred and forty-two patients were eligible for inclusion in the study and received the intervention.

Criteria for eligibility to participate in the study

Detailed criteria for inclusion were English-speaking adults admitted to the inpatient psychiatric facility, in the age group of 18 to 65 years, without discrimination for ethnic background, sex, or underlying psychiatric diagnosis. Individuals had to reside in the catchment area at the time of admission. The individuals of interest also were admitted on involuntary status. Participants had to have a working phone number. If a patient declined to participate, or were not reachable by phone, they were not included in the study but instead were considered part of the control group receiving the standard of care discharge. 

Detailed study procedure 

The purpose of the post discharge phone call program was to identify possible issues and connect the patient with the proper resources before these issues resulted in readmission. Ensuring adequate follow-up and medication adherence were identified as key issues that could arise early in the post-discharge period. July of 2019 was the first month of completed phone calls. Three psychiatrists made the phone calls each week. The calls were made three days per week when the psychiatrist was on service. Each psychiatrist received a daily administrative list of the discharged patients for that day, which guided their calls for the week. The patients each received two phone call attempts within 72 hours of discharge. Each psychiatrist followed a script using open-ended questions to address issues commonly associated with psychiatric readmission. The script was created based on a literature review of commonly identified reasons for psychiatric readmission and approved by the GIRB. The questions addressed the patient’s social supports, outpatient follow-up appointments, and medications. More specifically, the discharge instructions regarding the use of medication, ability to fill the prescription, names and information of two support sources, and the details of the patient’s follow-up appointments were directly addressed in each call. A triage algorithm guided the process if the patient experienced a specific problem. In the case a patient reported active suicidality, emergency services would be dispatched to the patients location. Weekly meetings to discuss any issues with making the phone calls, problems with the phone script, and changes to the script were performed as needed throughout the 12-month period.

Data collection

All patient information was obtained from the electronic medical record (EMR) and transferred to a database. This information was updated on a daily basis to determine if the call had been made, if the patient or caregiver was reached, and the result of the call intervention. Billing data were used to capture all admissions and readmissions during the study period. For patients with two or more readmissions within a 30-day period we included only the initial encounter and the first readmission. 

Statistical analysis 

We categorized our patients into two groups: those who met the criteria and received the post-discharge phone call, and those who did not receive the post-discharge phone call but otherwise met criteria for inclusion in the study. The data were analyzed using a Pearson's Chi-Square test. We used an alpha level of 0.05 for all statistical tests. A total percent readmission rate was calculated for the intervention group with an associated p-value. A 95% CI was also calculated for the average readmission rate in the intervention group. 

## Results

Readmissions within 30-days were considered early readmissions and thus had an overall negative outcome for both the patient and the healthcare system via costs accrued. The total average readmission rate for all patients admitted to the STCF was 9.9% (95% CI 5.9-12.1%) during the intervention year when compared to the previous year’s average of 13.3%, (P = 0.004). The total readmissions per month before and during the intervention are shown in Table 1. 

**Table 1:** Total readmission comparison by month and total for the study duration

Control	Percent (%)	Intervention	Percent (%)	P-Value
July 2018	15.0	July 2019	12.0	0.458
August 2018	19.0	August 2019	8.0	0.007
September 2018	13.0	September 2019	9.0	0.285
October 2018	17.0	October 2019	10.0	0.111
November 2018	19.0	November 2019	10.0	0.051
December 2018	10.0	December 2019	10.0	1.000
January 2019	11.0	January 2020	11.0	0.995
February 2019	11.0	February 2020	8.0	0.430
March 2019	7.0	March 2020	6.0	0.759
April 2019	14.0	April 2020	17.0	0.561
May 2019	13.0	May 2020	12.0	0.821
June 2019	10.0	June 2020	9.0	0.790
Total	13.3%	Total	9.9%	0.004

## Discussion

This study aimed to reduce readmission rates by providing additional support after discharge from a psychiatric hospital. Data from previous studies suggest patients who receive continuous follow-up are less likely to be hospitalized and have reduced readmission rates [1]. By addressing the commonly identified issues patients face post-discharge, there is potential to reduce decompensation and readmission. In patients discharged, follow-up with psychiatry appointments, social support networks, and medication management are considered to be common factors that can lead to readmission. During follow-up calls, many patients reported improved understanding of discharge medications and follow-up plans.

One study in Japan explained that follow-up systems help patients who show insidious symptoms and more serious behavioral symptoms [4]. Post-discharge interventions that include telephone calls provided a link between hospitalization and outpatient treatment for the patient [5]. Shepperd et al. concluded that many psychiatric patients are from low-income backgrounds with poor social support and thus, a close partnership is critical for discharge planning and care coordination [5]. 

This study’s primary outcome was to evaluate whether telephone follow-up reduced readmission rates. Few studies have looked at the involuntary readmission rates as a primary outcome. Although readmissions are affected by a variety of factors that are complex in nature, including bed availability, resources, community acceptance, and discharge policies [6], the implementation of telephone follow-up is a relatively simple tool to support patients. In psychiatry, many of our patients admitted to the inpatient unit have socio-economic issues that reduce their access to quality care. Some have suggested that 30-day readmission is not a valid marker of quality of care [7]. One such review concluded that readmission rates are a promising quality indicator, but several methodological concerns need to be addressed when using it to assess performance [8]. 

One area that we were unable to explore but which may provide additional value is the use of a text messaging service to provide the same information. Most patients have access to a smart device and may prefer to receive follow-up information in this manner. One study looked specifically at appointment reminders received via text message to reduce the 30-day readmission rate to inpatient psychiatric hospitals. They concluded that appointment reminders received as a letter, text message, or phone call may decrease 30-day readmission rates [9]. The average 30-day readmission rate prior to implementation was 10% and after implementation, the average readmission rate was 9% [9]. Our data indicate that post-discharge phone calls with more targeted objectives resulted in an additional reduction in 30-day readmission (total percent reduction in readmission 3.4%). 

Readmissions during COVID-19 months

At the end of 2019, a novel coronavirus was identified as the cause of a number of pneumonia cases in Wuhan, Hubei, China. The World Health Organization designated the disease Coronavirus Disease 2019 (COVID-19). It rapidly spread around the world with more than 20 million confirmed cases. COVID-19 led to isolation and quarantine, which required changes in the delivery of health care that may have impacted adverse mental health outcomes [10]. Research suggests that there was a reduction in psychiatric admissions during the early stages of the lockdown period, with admissions rates in the post-lockdown period increasing to pre-pandemic levels [11]. In New Jersey, the lockdown period lasted from March 16 to June 9, 2020. The total number of admissions during the COVID-19 lockdown period compared to 2019 admissions in the same month is shown in (Figure 1). 

**Figure 1:** Total number of admissions during COVID-19 lockdown period (orange) compared to 2019 (blue)

This study was ongoing at the start of the COVID-19 pandemic. Data were collected regarding the total admissions and readmission status of all psychiatric patients during the peak COVID-19 months of March to June 2020. The number of total admissions was higher in March, April, and May of 2019 but similar for the month of June. Of note, the readmission rates in 2020 during the lockdown period as compared to 2019 were similar and higher in the case of April 2020 than the readmission rate in 2019. The reduced number of admissions may have impacted the readmission results during these months. This could result in decreased readmission rates for several reasons including fear of infection with COVID-19. 

A comparative study of access to inpatient psychiatric care during COVID-19 identified patients at risk for inpatient admission during the COVID-19 lockdown period. The authors concluded that patients separated from their significant other, and those with a substance use disorder were more likely to seek inpatient treatment than others [12]. It may be valuable to reanalyze the data during the lockdown period to determine if similar factors contributed to inpatient admission.

Limitations include selection bias due to conducting the study at a single-site hospital. Other limitations include manpower, short duration of follow-up, and small sample size. Manpower was a significant issue for this study. Phone calls were made by resident physicians in addition to their normal clinical duties. A significant amount of time and energy is required to organize the discharge lists and make the phone calls within the 72-hour time window. A minimum of one to two hours per day were spent by each resident involved in this study performing these tasks over the course of the year. It would be helpful for hospital systems to have a dedicated person to make these calls and maintain the discharge list, although the cost may be a prohibiting factor. The sample size was fairly small for this type of study. It may be beneficial to expand the inclusion criteria or simply make a phone call to all patients discharged from the inpatient unit to increase the sample size and power of the study. The comparison group is also a limitation. The control group was people who would have qualified for the study but did not participate due to lack of access to a phone, or lack of general interest in participating. Since this could have affected participation, it may be a possible confounding factor. 

## Conclusions

This study’s primary outcome was to evaluate the utility of post-discharge phone calls as a method to reduce all-cause 30-day readmission. More than half the patients were more likely to follow up with their appointment and avoid readmission. The study population was considered severely mentally ill at the time of admission and thus would benefit from the improved transition of care after discharge compared to standard discharge procedures. This study demonstrated that post-discharge phone calls positively impacted readmission rates to a community-based inpatient psychiatric care facility. Programs would benefit from improving their ability to perform phone outreach after discharge, with designated callers trained to administer a script tailored to known areas of readmission risk. 
